The article "Imbalance of the intestinal virome and altered viral-bacterial interactions caused by a conditional deletion of the vitamin D receptor" was published in 2021. Journal: Gut Microbes.

# Imbalance of the intestinal virome and altered viral-bacterial interactions caused by a conditional deletion of the vitamin D receptor

**DOI:** 10.1080/19490976.2021.1957408

**Published:** 2021-08-10

**Authors:** Jilei Zhang, Yongguo Zhang, Yinglin Xia, Jun Sun

**Affiliations:** a Division of Gastroenterology and Hepatology, Department of Medicine, University of Illinois at Chicago, Chicago, IL, USA; b Department of Microbiology and Immunology, University of Illinois at Chicago, Chicago, IL, USA; c Department of Medicine, University of Illinois Cancer Center, University of Illinois at Chicago, Chicago, IL, USA; d Jesse Brown VA Medical Center Chicago, IL, USA

**Keywords:** (5-10): myeloid cells, microbiome, metabolites, nod, pattern recognition receptors, paneth cells, TLR

## Abstract

Vitamin D receptor (VDR) deficiency is associated with cancer, infection, and chronic inflammation. Prior research has demonstrated VDR regulation of bacteria; however, little is known regarding VDR and viruses. We hypothesize that VDR deficiency impacts on the intestinal virome and viral-bacterial interactions. We specifically deleted VDR from intestinal epithelial cells (VDR^ΔIEC^), Paneth cells (VDR^ΔPC^), and myeloid cells (VDR^ΔLyz^) in mice. Feces were collected for shotgun metagenomic sequencing and metabolite profiling. To test the functional changes, we evaluated pattern recognition receptors (PRRs) and analyzed microbial metabolites. *Vibrio* phages, *Lactobacillus* phages, and *Escherichia coli* typing phages were significantly enriched in all three conditional VDR-knockout mice. In the VDR^ΔLyz^ mice, the levels of eight more virus species (2 enriched, 6 depleted) were significantly changed. Altered virus species were primarily observed in female VDR^ΔLyz^ (2 enriched, 3 depleted) versus male VDR^ΔLyz^ (1 enriched, 1 depleted). Altered alpha and beta diversity (family to species) were found in VDR^ΔLyz^. In VDR^ΔIEC^ mice, bovine viral diarrhea virus 1 was significantly enriched. A significant correlation between viral and bacterial alterations was found in conditional VDR knockout mice. There was a positive correlation between *Vibrio* phage JSF5 and *Cutibacterium acnes* in VDR^ΔPC^ and VDR^ΔLyz^ mice. Also, there were more altered viral species in female conditional VDR knockout mice. Notably, there were significant changes in PRRs: upregulated TLR3, TLR7, and NOD2 in VDR^ΔLyz^ mice and increased CLEC4L expression in VDR^ΔIEC^ and VDR^ΔPC^ mice. Furthermore, we identified metabolites related to virus infection: decreased glucose in VDR^ΔIEC^ mice, increased ribulose/xylulose and xylose in VDR^ΔLyz^ mice, and increased long-chain fatty acids in VDR^ΔIEC^ and VDR^ΔLyz^ female mice. Tissue-specific deletion of VDR changes the virome and functionally changes viral receptors, which leads to dysbiosis, metabolic dysfunction, and infection risk. This study helps to elucidate VDR regulating the virome in a tissue-specific and sex-specific manner.

The article "Imbalance of the intestinal virome and altered viral-bacterial interactions caused by a conditional deletion of the vitamin D receptor" was published in 2021. Journal: Gut Microbes.

## Introduction

During the pandemic, the correlation of vitamin D status and risk of coronavirus disease 2019 (COVID-19) are inspiring the heath-workers and researchers for prevention and treatment of this deathful diseases.^1^^, 2^ Actually, the role of vitamin D in viral infection is not a new topic. Vitamin D acts through the VDR, an ancient nuclear receptor and a transcription factor highly conserved in mammals.^3,4^ The expression level of VDR is very high in the small intestine and colon and plays an important role in local and systemic immunity, host defense, and host-microbial interactions.^5–11^ Vitamin D/VDR deficiency is not only associated with various digestive diseases, but also plays an important role in viral infection, including influenza infections,^12–16^ Epstein-Barr virus infection,^17^ varicella-zoster virus infection,^18^ cytomegalovirus infection,^17^ and hepatitis C virus infection.^19^ An epidemiological study showed an inverse association between vitamin D levels in the serum and infections of the upper and lower respiratory tracts.^20^ Vitamin D deficiency also contributes to the pathogenesis of HIV infection by negatively modulating innate and adaptive immune responses.^21,22^ At the gene level, a meta-analysis determined that the *VDR* gene polymorphism *FokI* is consistently associated with host susceptibility to infection by respiratory syncytial virus.^23^ Gene variation in VDR was also reported to correlate with persistent hepatitis B infection in clinical patient samples.^24^ Consistent with the epidemiological data, activation of the vitamin D/VDR pathway in response to respiratory syncytial virus infection occurs in lung cells via TLR3 signaling, which results in the induction of the CAMP gene.^25,26^ These observations highlighted the critical role in host defense by altering inductions of antimicrobial peptides and inflammatory cytokines in response to virus infection.

The human microbiota is consisted of bacteria, viruses, fungi, multicellular parasites and archaea. The virome is a collection of nucleic acids. Both RNA and DNA that compose the viral community associated with a particular ecosystem of microbiota. The virome includes viruses that infect host cells, virus-derived elements in the genome, and viruses that infect the broad array of other types of microorganisms that inhabit the host.^27^ The virome includes eukaryotic viruses, endogenous retroviruses, bacterial viruses (i.e., bacteriophages), and archaeal viruses and is one of the least understood components of the microbiota.^28,29^ Fecal virome was involved in many diseases using samples from both human patients and mouse model, such as colitis and diabetes.^30–34^ Dysbiosis of the microbiome not only leads to intestinal inflammatory and infectious diseases but also to diseases beyond the gastrointestinal tract.^5,35^ Moreover, dysbiosis of intestinal microbiota could influence internally through interaction and metabolites, such as bacteriophages and bacteria.^36^ At present, we are beginning to understand the influence of VDR on microbial homeostasis, which is critical in various diseases.^5,37–40^ However, the effects and mechanisms of VDR on the virome have not been fully elucidated.

The article "Imbalance of the intestinal virome and altered viral-bacterial interactions caused by a conditional deletion of the vitamin D receptor" was published in 2021. Journal: Gut Microbes.

In this study, we hypothesize that host factors (e.g., VDR status in specific tissues) are regulators of the intestinal virome, virus-bacterial interactions, and microbial metabolites. We conditionally deleted VDR from intestinal epithelial cells (VDR^ΔIEC^), Paneth cells (VDR^ΔPC^), and myeloid cells (VDR^ΔLyz^) of mice. Fecal samples from VDR knockout mice and their control VDR^loxp^ mice were collected for microbial DNA extraction, shotgun metagenomic sequencing, and metabolite analysis. Specifically, we used these novel animal models and statistical and bioinformatic tools/models to understand the interactions between host genetic factors and aspects of metabolites and intestinal microbiome, including bacteria and viruses. From a functional perspective, we investigated the virus infection-associated metabolites and virome-related PRRs of colonic epithelial cells. Understanding the role of VDR in altering the multi-kingdom aspects of the microbiome, including bacteria and viruses, may help to elucidate the mechanisms by which VDR regulates microbial homeostasis in terms of health and disease.

## Results

### Overall virome community composition in conditional VDR knockout mice

In all 40 fecal samples in 4 groups (each group had 10 mice equally 5 male and 5 female mice for the conditional VDR knockout groups and the control VDR^LoxP^ group had 7 female and 3 male mice), totally 4,048 viral species were identified. Distinct viral compositions and communities, which differed in both diversity and composition, were present between the control mice (VDR^LoxP^) and the conditional VDR knockout mice (VDR^ΔIEC^, VDR^ΔPC^, and VDR^ΔLyz^ mice) (Figure 1). We presented the 10 most abundant viral species for individual samples in each group (Figure 1). The most abundant species in the groups were *Vibrio* phage JSF5, *Vibrio* phage JSF6, BVDV-1 (Bovine Viral Diarrhea Virus 1), *Escherichia coli* O157 typing phage 7, human alphaherpesvirus 1, *Lactobacillus* prophage Lj771, influenza A virus, *Lactobacillus* phage KC5a, and viruses *incertae sedis* unidentified phage (Figure 1a). When individually analyzing the species, it was apparent that *Vibrio* phages JSF5 and JSF6 were significantly more abundant in all three VDR KO mouse models compared to control VDR^LoxP^ mice. *Escherichia coli* O157 typing phage 7 was found to be significantly more abundant in VDR^ΔPC^ mice, compared to the control mice. Meanwhile, *Lactobacillus* phage phiadh was considerably less abundant in VDR^ΔLyz^ mice compared to control VDR^LoxP^ mice (Figure 1b) (*P* < .01).

The article "Imbalance of the intestinal virome and altered viral-bacterial interactions caused by a conditional deletion of the vitamin D receptor" was published in 2021. Journal: Gut Microbes.

**Figure 1.** Altered taxa abundance of viruses in feces of the three conditional VDR-knockout (VDR^ΔIEC^, VDR^ΔPC^ and VDR^ΔLyz^) and control VDR^LoxP^ mice. (a) Relative viral abundance at the species level (family/f_; s_; the unidentified species were named with super level and other) is shown with the top 10 species, and less abundant species were grouped as “others”. Species were colored using the key as listed on the right side of the figure. Each bar represents an individual mouse. n = 10 each group. VDR^LoxP^: 7 females & 3 males; VDR-knockout groups: 5 females & 5 male per group. (b) The virus differential abundance at count per million of the top 10 species in four studied mouse genotypes are illustrated with different colors. Statistical analysis in each group was compared to control VDR^LoxP^ mice. Mean ± SD, n = 10 per group; ** *P*-value < 0.01, * *P*-value < 0.05, Kruskal–Wallis test by ranks

## Altered diversity of the virome in conditional VDR knockout mice

Shannon diversity is commonly used to characterize species diversity in a community.^41^ We found that the Shannon diversity at the viral species level was significantly lower in VDR^ΔIEC^, VDR^ΔPC^, and VDR^ΔLyz^ mice than in VDR^LoxP^ control mice (*P* = .05, *P* = .05, and *P* = .04, respectively) (Figure 2a).

**Figure 2.** Alpha and beta diversity of viral abundance in feces from the four genotypes of mice. (a) Violin plots presenting alpha diversity measurements. The Shannon diversity index was used to determine the alpha diversity differences of intestinal viruses between the control group (VDR^LoxP^) and conditional VDR-knockout mice (VDR^ΔIEC^, VDR^ΔPC^ and VDR^ΔLyz^), n = 10 each group. *P*-value as indicated above the plots. (b) The principal coordinates analysis (PCoA) plot of the mouse fecal samples was produced to inspect the homogeneity multivariate dispersions. The samples collected from different mouse genotypes are colored in the illustration, n = 10 per group. (c) Plots of between- and within-means Bray-Curtis dissimilarity. Analysis of similarity (ANOSIM) was performed to compare between dissimilarity and within dissimilarity of VDR^LoxP^, VDR^ΔIEC^, VDR^ΔPC^ and VDR^ΔLyz^ mice based on Bray-Curtis dissimilarity, n = 10 each group

The Bray-Curtis dissimilarity index was used in this study to measure the dissimilarities of samples.^42^ We first performed PCoA and found viral dissimilarities between conditional VDR knockout mice and control mice (Figure 2b). VDR^ΔIEC^ mice partially overlapped with control VDR^LoxP^ mice, whereas VDR^ΔPC^ and VDR^ΔLyz^ mice were completely separated from VDR^LoxP^ mice. Thus, PCoA suggested that the sample dissimilarities among these four groups and the group differences can explain a total of 37.2% (29.3% + 7.9%) of the variations among the animals.

The article "Imbalance of the intestinal virome and altered viral-bacterial interactions caused by a conditional deletion of the vitamin D receptor" was published in 2021. Journal: Gut Microbes.

Next, we performed nonparametric PERMANOVA to evaluate whether VDR status impacts the overall intestinal viral profile. The sequential test “Group and Gender” showed that the dissimilarities among groups were significantly different (*P* = .011). Because the overall dissimilarity among groups was significantly different, we performed a pairwise PERMANOVA and found that the Bray-Curtis dissimilarities of viruses of the VDR^ΔIEC^, VDR^ΔPC^, and VDR^ΔLyz^ mice had significantly different dissimilarities in the VDR^LoxP^ mice. Furthermore, the differences in dissimilarity among groups were confirmed by ANOSIM (analysis of similarity), where the rank dissimilarities between and within groups were significantly different (*P* = .001). VDR^ΔIEC^, VDR^ΔPC^, and VDR^ΔLyz^ mice had higher dissimilarities (i.e., lower similarity) than VDR^LoxP^ mice (Figure 2c).

### Altered abundance of the virome in conditional VDR knockout mice

We observed that a total of 12 viral species were differential in the conditional VDR knockout mice compared to the control VDR^LoxP^ mice, of which 6 had q-values <0.001, 2 had q-values <0.01 and 4 had q-values <0.05 (Figure 3a). The log-ratio of fold change with significant differences (q < 0.05) is shown with colored histograms (Figure 3). There were two enriched viral species in the comparison of VDR^ΔIEC^/VDR^LoxP^, *Vibrio* phage JSF5 (q < 0.001) and bovine viral diarrhea virus 1 (q < 0.05), and one enriched viral species in the comparison of VDR^ΔPC^/VDR^LoxP^, *Vibrio* phage JSF5 (q < 0.01). *Vibrio* phage JSF5 was more abundant in both VDR^ΔIEC^ and VDR^ΔPC^ mice, whereas enriched BVDV1 was only found in VDR^ΔIEC^ compared with the other groups (Figure 3a). For the comparison of VDR^ΔLyz^ and VDR^LoxP^, nine virus species were found to be significantly altered (5 with a q value <0.001, 1 with q < 0.01, and 3 with a q value <0.05). Of these species, three were enriched (*Vibrio* phage JSF5, bovine viral diarrhea virus 1 and *Vibrio* phage JSF6), while six were depleted (*Lactobacillus* prophage phiadh, Cherry green ring mottle virus, *Lactobacillus* phage KC5a, avian avulavirus 1, *Mycobacterium* virus Phayonce, and one unidentified species in the *Podoviridae* family) (Figure 3a).

The article "Imbalance of the intestinal virome and altered viral-bacterial interactions caused by a conditional deletion of the vitamin D receptor" was published in 2021. Journal: Gut Microbes.

**Figure 3.** Differential analysis of viral genes in the feces of mice of four genotypes. (a) Log_2_-fold changes (FC) of viral species with a *P*-value ≤ 0.05 are shown by increasing (red) or decreasing (blue) in three pairwise comparisons: VDR^ΔIEC^/VDR^LoxP^, VDR^ΔPC^/VDR^LoxP^ and VDR^ΔLyz^/VDR^LoxP^, n = 10 each group. *** indicates q value (FDR-corrected *p*-value) <0.001, ** indicates q-value < 0.01, * indicates q-value < 0.05, # indicates q-value < 0.1. (b) Viral species with q-values ≤0.05 in both female and male pairwise comparisons are shown with fold-changes (logFCs) and q-values in three comparisons between the conditional VDR knockout groups (VDR^ΔIEC^, VDR^ΔPC^, and VDR^ΔLyz^) and control mice (VDR^LoxP^). Both fold-change and q-value were colored using the key as listed on the right side of the figure, n = 10 each group

### Sex-based differences in the gut virome altered by VDR status

To investigate the impact of sex on the alteration of the virome community in the intestines of the studied mice, we illustrated significantly different virus species abundances in male and female mice with logarithmic fold-changes and q-values (Figure 3b). In our study, both male and female mice were included in all the investigated groups, VDR^LoxP^: male n = 3 and female n = 7; VDR^ΔIEC^: male n = 5 and female n = 5; VDR^ΔPC^: male n = 5 and female n = 5; VDR^ΔLyz^: male n = 5 and female n = 5. Seven species were detected to be significantly altered in the female VDR^ΔIEC^/VDR^LoxP^ comparison but not when comparing males of the same two groups, the altered species included 2 enriched species, *Vibrio* phages JSF5 and BVDV1, and 5 depleted species, *Lactobacillus* prophage phiadh, *Lactobacillus* prophage KC5a, *Lactobacillus* prophage Lj771, macacine alphaherpesvirus 1 and Catovirus CTV1. However, only *Vibrio* phage JSF5 was enriched in female VDR^ΔPC^ mice compared to control VDR^LoxP^ mice (Figure 3b), which is the same as in the group-factor analysis. Five species in the female VDR^ΔLyz^/VDR^LoxP^ comparison were found to be significantly differential (q < 0.05), including 2 enriched species: *Vibrio* phage JSF5 and bovine viral diarrhea virus 1, and 3 depleted species, *Lactobacillus* prophage phiadh, Cherry green ring mottle virus and *Lactobacillus* prophage KC5a, while in males, only *Vibrio* phage JSF5 was enriched and only *Lactobacillus* prophage phiadh was depleted (Figure 3b). Overall, more altered viral species in all conditional VDR knockout mice were found in the female mice than in male mice, which indicated the impact of VDR status on sex differences.

The article "Imbalance of the intestinal virome and altered viral-bacterial interactions caused by a conditional deletion of the vitamin D receptor" was published in 2021. Journal: Gut Microbes.

### VDR deletion led to significantly enriched Vibrio phages

*Vibrio* phages target *Vibrio cholerae* bacteria, which can secrete cholera toxin and cause watery diarrhea in patients and mouse models.^43–46^ In this study, we found a markedly enriched abundance of *Vibrio* phage JSF5 and *Vibrio* phage JSF6 in VDR^ΔIEC^, VDR^ΔPC^, and VDR^ΔLyz^ mice compared with control VDR^LoxP^ mice (Figure 1). Moreover, differential analysis found that *Vibrio* phage JSF5 was significantly enriched in all three conditional VDR-knockout mice (q < 0.01) compared to the control mice, and *Vibrio* phage JSF6 was also more enriched in VDR^ΔLyz^ mice in comparison to VDR^LoxP^ mice (q < 0.01) (Figure 3). When the sex factor was included in the analysis, the fold-changes of *Vibrio* phage JSF5 were found to be significant in both female and male VDR^ΔLyz^ mice but only in female VDR^ΔIEC^ and VDR^ΔPC^ mice (Figure 3).

### Altered bacterial abundance in conditional VDR knockout mice

We reasoned that the abundance of bacteria in the intestines of the mice should be altered based on our findings of the dysbiosis of bacteriophages. In this study, we found that *Vibrio cholerae*, the host of *Vibrio* phage JSF5 and *Vibrio* phage JSF6, which were largely enriched in conditional VDR knockout mice (Figure 1b), was detected at low concentrations in knockout mice compared with control mice (Figure 4a). Significantly lower abundance of this bacterium was found in VDR^ΔLyz^ mice, which matches the finding that both *Vibrio* phage JSF5 and *Vibrio* phage JSF6 were enriched in VDR^ΔLyz^ mice. A similar situation was also found in *Lactobacillus gasseri*, the bacterial host of *Lactobacillus* prophage phiadh and *Lactobacillus* prophage KC5a (Figure 1b; Figure 4a). Furthermore, as the target host of *Escherichia coli* O157 typing phage 7, *E. coli* bacterial abundance was found altered in a opposite way as phage species in the mice studied here (Figure 1b; Figure 4a). The altered bacterial abundance in the microbial community supports our findings of virome changes.

**Figure 4.** Altered bacterial abundance and correlations with viral alteration. (a) Bacterial species related to the altered bacteriophages were shown with bacterial differential abundance at count per million, including *Vibrio cholerae, Lactobacillus gasseri* and *Escherichia coli*. Mean ± SD, n = 10 per group; Kruskal-Wallis test. (b) Log_2_-fold changes (FCs) of bacterial species with q-values ≤ 0.1 are shown by increasing (red) or decreasing (blue) in three pairwise comparisons: VDR^ΔIEC^/VDR^LoxP^, VDR^ΔPC^/VDR^LoxP^ and VDR^ΔLyz^/VDR^LoxP^, n = 10 each group. *** indicates q value (FDR-corrected *p*-value) <0.001, ** indicates q < 0.01, * indicates q < 0.05, # indicates q < 0.1. (c) Correlation matrix of bacteria and viruses in the feces of conditional VDR knockout mice. The correlation of viral (vertical) and bacterial (horizontal) species with a q-value ≤0.05 in differential analysis was analyzed using the Hmisc package in R. The positive-correlation (red background) and negative-correlation (green background) values are shown in the map. *** indicates *P* < .001, * indicates P ≤ 0.05, n = 10 each group

To further evaluate the altered bacterial composition, we showed the altered bacterial species with q-values <0.1 in differential analysis in our three mouse models (Figure 4b). We found that *Haemophilus ducreyi* and *Mesorhizobium huakuii* were significantly depleted in VDR^ΔIEC^ mice compared with control VDR^LoxP^ mice (Figure 4b). Meanwhile, five bacterial species were significantly depleted, and three bacterial species were significantly enriched in VDR^ΔPC^ mice, compared with the control. These depleted species were *Haemophilus ducreyi Kushneria konosiri, Microbacterium* sp. LKL04, *Isosphaera pallida*, and *Actinomyces radingae*. Three enriched bacterial species were *Bacteroides uniformis, Faecalibaculum rodentium*, and *Cutibacterium acnes* (q < 0.01. Figure 4b). Furthermore, we found that nine bacterial species were significantly depleted, and three bacterial species were enriched in VDR^ΔLyz^ mice. These depleted bacterial species were *Bifidobacterium pseudolongum, Bifidobacterium choerinum, Bifidobacterium animalis, Bordetella pseudohinzii, Haemophilus ducreyi, Clostridium perfringens, Streptomyces peucetius*, and *Bacteroides acidifaciens*. The three enriched bacterial species were *Ralstonia solanacearum, Chroococcidiopsis thermalis*, and *Cutibacterium acnes* (Figure 4b). The less abundant *Haemophilus ducreyi* is a gram-negative bacterium and causative agent of genital ulcer disease chancroid^47^ and was detected in the three conditional VDR knockout mice. Similar to viruses, more bacterial species were enriched (7 in total) or depleted (24 in total) in VDR^ΔPC^ and VDR^ΔLyz^ mice compared to the control mice (Figure 4b).

The article "Imbalance of the intestinal virome and altered viral-bacterial interactions caused by a conditional deletion of the vitamin D receptor" was published in 2021. Journal: Gut Microbes.

### Correlation of viral and bacterial alterations in conditional VDR KO mice

Bacteria and viruses are essential for protective, metabolic, and physiological functions.^48^ We found that the viral (consisting mostly of bacteriophages) and bacterial species abundances were altered in conditional VDR KO mice. To investigate the interactions between bacteria and viruses, we performed a correlation analysis of viruses and bacteria. All the bacterial and viral species with significant fold changes in the differential analysis (q < 0.05) were included in the correlation analysis (Figure 4c and Supplement Table 1).

**Table 1.** Primers for real-time PCR used in this study

Primer	Gene	Sequence (5ʹ – 3ʹ)	Reference
TLR3-F	*tlr3*	GTGAGATACAACGTAGCTGACTG	^49^
TLR3-R	*tlr3*	TCCTGCATCCAAGATAGCAAGT	
TLR7-F	*tlr7*	ATGTGGACACGGAAGAGACAA	^50^
TLR7-R	*tlr7*	GGTAAGGGTAAGATTGGTGGTG	
NOD1-F	*nod1*	GAAGGCACCCCATTGGGTT	^51^
NOD1-R	*nod1*	AATCTCTGCATCTTCGGCTGA	
NOD2-F	*nod2*	CAGGTCTCCGAGAGGGTACTG	^51^
NOD2-R	*nod2*	GCTACGGATGAGCCAAATGAAG	
NLRp6-F	*nlr6*	CTCGCTTGCTAGTGACTACAC	^52^
NLRp6-R	*nlr6*	AGTGCAAACAGCGTCTCGTT	
CLEC4L-F	*clec4l*	CCTGAACACAAGTGCTGGTTA	This study
CLEC4L-R	*clec4l*	CACATCGTTCCCAATCTTGGT	

In VDR^ΔIEC^ mice, bovine viral diarrhea virus 1 was significantly negatively correlated with the bacteria *Mesorhizobium huakuii* (correlation coefficient (r) = −0.63; *P* = .05) (Figure 4c). *M. huakuii* induces the formation of nitrogen-fixation nodules on its host plant *Astragalus sinicus* and has been assigned to a new biovariety based on its host range and taxonomic characteristics. ^49^ *M. huakuii* isolates were also found to have endotoxic activity against lipopolysaccharides.^53^ In VDR^ΔPC^ mice, the *Vibrio* phage JSF5 was dramatically positively correlated with the bacteria *Cutibacterium acnes* (r = 0.98; *P* < .0001) (Figure 4c). *Cutibacterium acnes*, formerly known as *Propionibacterium acnes*, is an anaerobic, aerotolerant, bacillus-shaped bacterium. It is ubiquitously found as a commensal on the surface of skin in areas rich in oleic and palmitic acids.^54^ Moreover, variable results for the association between *C. acnes* and ulcerative colitis were found.^55^ In VDR^ΔLyz^ mice, 11 pairs of virus-bacteria were found to be significantly correlated (5 positive-correlation, 6 negative-correlation), including *Vibrio* phage JSF5 and *Bordetella pseudohinzii* (r = 0.65; *P* = .04), *Vibrio* phage JSF5 and *Cutibacterium acnes* (r = 0.68; *P* = .03), bovine viral diarrhea virus 1 and *Bifidobacterium animalis* (r = −0.64; *P* = .05), bovine viral diarrhea virus 1 and *Haemophilus ducreyi* (r = 0.65; *P* = .04), bovine viral diarrhea virus 1 and *Bacteroides acidifaciens* (r = −0.66; *P* = .04), bovine viral diarrhea virus 1 and *Bifidobacterium* sp. (r = −0.66; *P* = .04), Lactobacillus phage phiadh and *Clostridium perfringens* (r = −0.71; *P* = .02), *Vibrio* phage JSF6 and *Bifidobacterium animalis* (r = −0.67; *P* = .03), *Vibrio* phage JSF6 and *Ralstonia solanacearum* (r = 0.65; *P* = .04), *Vibrio* phage JSF6 and *Haemophilus ducreyi* (r = 0.75; *P* = .01), and *Podoviridae* (family level) and *Chroococcidiopsis thermalis* (r = −0.75; *P* = .01) (Figure 4c). In addition, we found a positive correlation between *Vibrio* phage JSF5 and *Cutibacterium acnes* in VDR^ΔPC^ mice and VDR^ΔLyz^ mice. Taken together, these data indicate the critical role of viral and bacterial interactions in intestinal microbial homeostasis with the support of VDR.

The article "Imbalance of the intestinal virome and altered viral-bacterial interactions caused by a conditional deletion of the vitamin D receptor" was published in 2021. Journal: Gut Microbes.

### VDR status altered the expression of PRRs in colonic epithelial cells

To examine the impact of virome dysbiosis, virus-related receptors in the colon were evaluated (Figure 5). TLR3 and TLR7 are transmembrane PRRs located in endosomes that recognize nucleic acids and mediate cell extrinsic virus recognition.^56^ We observed that expression of TLR3 and TLR7 was upregulated in the conditional VDR knockout mice compared with the control mice, with a significant difference in the VDR^ΔLyz^ group vs. the control group (*P* < .05) (Figure 5).

**Figure 5.** Altered pattern recognition receptors in the colon of VDR conditional knockout mice. Expression of virus translocation-related PRRs in the intestine, including TLR3, TLR7, NOD1, NOD2, NLRP6, and CLEC4L, was performed with colon epithelial cells using real-time quantitative PCR. Mean ± SD, n = 3; ** *P*-value < 0.01, * *P*-value < 0.05, one-way ANOVA

NLRs characterized by the presence of a conserved NOD motif, comprise a large receptor family, including NOD1, NOD2, and NLRPs.^57,58^ NLRs are activated not only in response to viruses but are also important modulators of other virus sensing pathways.^56^ Here, we observed upregulated expression of NOD1 and NLRP6 and significantly increased NOD2 RNA in VDR^ΔLyz^ mice compared with control VDR^LoxP^ mice (*P* < .05) (Figure 5). C-type lectin receptors (CLRs) also mediate cell-extrinsic sensing of specific viruses by binding viral glycans.^59^ Compared with the control VDR group, the expression of CLEC4L, one of the CLRs, was significantly upregulated in all three conditional VDR knockout mice, especially in VDR^ΔIEC^ and VDR^ΔPC^ mice (Figure 5). Overall, the significant alterations of PRRs in conditional VDR knockout mice suggest the influence of VDR on intestinal homeostasis and expression of PRRs.

### VDR status altered metabolites related to bacteriophage infection in feces

Microbiota-derived metabolites are chemical messengers that elicit a profound impact on host physiology. Thus, we investigated bacterial metabolites that are related to bacteriophage infection as reported before^36^ (Figure 6). We found that glucose in glycolysis pathway was significantly decreased in VDR^ΔIEC^ mice compared with the control (*P* < .05), while ribulose/xylulose and xylose were significantly increased in VDR^ΔLyz^ mice compared with the control (*P* < .05) (Figure 6a). Moreover, most of the long-chain fatty acids were significantly increased in both VDR^ΔIEC^ and VDR^ΔLyz^ female mice compared to control mice, while some fatty acids were only increased in VDR^ΔIEC^ mice. 10-Hydroxystearate, which was significantly changed after phage infection as reported before,^36,48^ was decreased in VDR^ΔLyz^ mice and increased in female VDR^ΔIEC^ mice compared to control mice (*P* < .05) (Figure 6b). Metabolic alterations of nucleotides were also detected in both conditional knockout mice, such as uridine in VDR^ΔIEC^ mice and 3-ureidoisobtyrate in VDR^ΔLyz^ mice (*P* < .05) (Figure 6c). Similarly, we observed amino acid alterations in the feces of conditional VDR knockout mice when compared to those of the control mice. For instance, we observed decreased phage infection-related serine in both VDR^ΔIEC^ and VDR^ΔLyz^ female mice and decreased cellular virus infection-related glutamine in VDR^ΔIEC^ and VDR^ΔLyz^ female mice compared to the control (Figure 6d).

The article "Imbalance of the intestinal virome and altered viral-bacterial interactions caused by a conditional deletion of the vitamin D receptor" was published in 2021. Journal: Gut Microbes.

**Figure 6.** Altered virus infection-related metabolites in the feces of VDR conditional knockout mice and controls. A heatmap of fold changes of metabolites related to virus infection (regular font) and bacteriophage infection (bold font) is shown in both male and female VDR^ΔIEC^, VDR^ΔPC^, VDR^ΔLyz^ and control mice (VDR^LoxP^) with different pathways, including carbohydrates (a), lipids (b), nucleotides (c) and amino acids (d). Mean ± SD, n = 5–10; * *P*-value indicated as the color bar on the right and together with the number inside the blocks, two-way ANOVA

## Discussion

In the current study, we found that conditionally deleted VDR from mouse intestinal epithelial cells, Paneth cells, and myeloid cells could significantly alter the virome profile and virome-bacterial interactions in the gut (summarized in Figure 7). Overall, the components of *Vibrio* phages, *Lactobacillus* phages, and *E. coli* typing phage in the gut were significantly altered in the conditional VDR knockout mice. The viral alteration was variable due to different VDR deletion, such as seven more virus species were significantly changed in VDR^ΔLyz^ mice, while BVDV1 was significantly enriched in VDR^ΔIEC^ mice compared to control mice. Meanwhile, a significant correlation between viral and bacterial alterations was found in conditional VDR knockout mice. For instance, a positive correlation between *Vibrio* phage JSF5 and *Cutibacterium acnes* in VDR^ΔPC^ and VDR^ΔLyz^ mice. Moreover, we found the gender difference in our VDR deficiency mouse model, which was supported by the greater alteration of viral abundance in female mice than in male mice. As we know, bacteriophages could modulate their hosts directly by affecting their mortality and horizontal gene transfer or indirectly by impacting target/host bacteria and hence may alter the microbiome.^60^ After conditionally deleting VDR, the virome and other aspects of the microbiota in the gut were changed, which further led to microbial dysbiosis. From a functional perspective, the significant changes in PRRs and metabolites related to infection suggest the influence of VDR on intestinal virus homeostasis.

The article "Imbalance of the intestinal virome and altered viral-bacterial interactions caused by a conditional deletion of the vitamin D receptor" was published in 2021. Journal: Gut Microbes.

**Figure 7.** Summary of animal models, groups, cellular changes, metabolites, and microbiome in the VDR conditional knockout mice. Three conditional VDR-knockout (VDR^ΔIEC^, VDR^ΔPC^, and VDR^ΔLyz^: 5 females & 5 male each group) and control VDR^LoxP^ mice (7 females & 3 males). n = 10 each group

One of primary goals of this study is to build an appropriate statistical method to analyze interactions among intestinal bacteria, phages, and virome. *Vibrio* phages JSF5 and JSF6 are organisms hosted by *Vibrio cholera*, which can secrete cholera toxin and cause watery diarrhea in patients.^43,44^ The *Lactobacillus* phages phiadh and KC5a are members of the viral family *Siphoviridae* and can preferentially infect the bacteria *Lactobacillus gasseri*, which is a common component of intestinal mucosae and plays an important role in modulating the gut immune system.^61^ These observations were consistent with our results that VDR deletion in myeloid cells had a more severe influence on the intestinal virome balance. Similarly, the interactions in the microbial community are important to maintain homeostasis and host health. For instance, viruses can bind to bacterial products (e.g., lipopolysaccharide or HBGA (human blood group antigen)-like substances), increase virome stability and protect virome from physical stresses.^62^ We also found that the *Lactobacillus* phage KC5a and *E. coli* O157 typing phage 7, which belong to the family *Myoviridae*, and *Lactobacillus* phage phiadh, which belongs to the family *Siphoviridae*, were altered in our conditional VDR knockout mouse models compared with the control mice. A study indicated that the Crohn’s disease (CD) susceptibility gene *ATG16L1* was phenocopied in mice infected with murine norovirus.^63–65^ Meanwhile, we have previously demonstrated that VDR transcriptionally regulates *ATG16L1*, and VDR status may be a determinant of Inflammatory Bowel Disease (IBD) risk through its actions on *ATG16L1*.^37,66^ However, these results may support a model in which bacteriophages contribute to the development of bacterial dysbiosis associated with IBD. Bacteriophages modulate their hosts directly by affecting their mortality and horizontal gene transfer and by further altering the components of the intestinal community and contributing to dysbiosis.^28^ The virome could be a candidate biomarker for human IBD^67^ because IBD were associated with a significant expansion of *Caudovirales* bacteriophages. The phage families of the *Caudovirales* order, including the *Siphoviridae, Myoviridae* and *Podoviridae*, were found to be altered in murine colitis and human IBD patients.^68^ Therefore, further studies are needed to elucidate the important and real role of the intestinal virome in the development and progression of IBD.

The article "Imbalance of the intestinal virome and altered viral-bacterial interactions caused by a conditional deletion of the vitamin D receptor" was published in 2021. Journal: Gut Microbes.

Our previous reports demonstrated that VDR could promote healthy microbial metabolites and a healthy microbiome to prevent obesity.^69^ Furthermore, it has been reported that increased serum 25(OH)D was associated with increased beneficial bacteria, such as *Parabacteroides*, which were suppressed in IBD patients and were altered in an obesity mouse model.^69,70^ We have reported that human *VDR* gene variation determines the abundance of *Parabacteroides*.^39^ In this study, we also found a decreased abundance of *Parabacteroides* in three VDR knockout mice (VDR^ΔPC^, VDR^ΔIEC^ and VDR^ΔLyz^) compared with VDR^LoxP^ controls. This further confirms the critical role of VDR in shaping the gut microbiome, including the eukaryotic virus and bacteriophages, at the genetic level.

Paneth cells play an integral role in shaping the microbiome and host defenses. The absence of VDR in Paneth cells impairs antimicrobial function, affects microbial assemblage, and increases susceptibility to colitis and infection.^37,71^ The altered virome in VDR^ΔPC^ mice further indicated the important role of VDR and Paneth cells in shaping the intestinal microbiome and secreting antimicrobial peptides or metabolites. Paneth cells may indirectly impact the intestinal microbiota or the outcome of a viral infection by adjusting the population of bacteria. Paneth cells also play a key role in host defense by sensing microorganisms through TLRs.^72^ It is clear from our data that VDR deficiency in Paneth cell could lead to viral dysbiosis, which may further result in a compromised epithelial barrier.^72^

Eukaryotic viruses, such as adenoviruses, hepatitis B virus, hepatitis C virus and human immunodeficiency virus,^73^ are also present in the intestinal virome of some individuals, which indicates the potential infectious capability of these eukaryotic viruses in the host. BVDV1 can infect mice and cause significant histopathological damage.^74^ The significantly increased abundance of intestinal BVDV1 in VDR conditional knockout mice suggested the importance of VDR in viral infection and survival inside the host. Furthermore, the association between vitamin D deficiency and the pathogenesis and course of HIV disease has also been recognized recently. Infants born from HIV-infected women with vitamin D deficiency are at an increased risk of infection and a decreased survival rate.^75^ In addition, the VDR polymorphism *FokI* was evaluated using a meta-analysis to be consistently associated with susceptibility to infection to respiratory syncytial virus.^23^

The article "Imbalance of the intestinal virome and altered viral-bacterial interactions caused by a conditional deletion of the vitamin D receptor" was published in 2021. Journal: Gut Microbes.

The innate immune response is nonspecific, is the first line of defense against infectious agents and initiates antigen presentation, including responses to viral infection. PRRs and related pathways involved in intestinal virus sensing, such as TLRs, are mainly mediated by cell-extrinsic virus recognition.^76^ We found significant alterations in PRRs, including upregulated expression of TLR3, TLR7 and NOD2 in VDR^ΔLyz^ mice and increased expression of CLEC4L in VDR^ΔIEC^ and VDR^ΔPC^ mice, suggesting the influence of VDR on intestinal virus homeostasis. Our data further suggest that the impacts of tissue-specific VDR deletion on intestinal receptors are different. For instance, VDR deletion in myeloid cells would significantly increase the expression of TLR3, TLR7 and NOD2, while VDR deletion in intestinal epithelial cells would more likely increase CLEC4L levels. TLRs are known to be affected by VDR in monocytes and epidermal keratinocytes.^12^ In mice administered an antiviral drug cocktail, the depletion of gut viral entities could increase susceptibility to Dextran sulfate sodium-induced colitis via TLR3 and TLR7 signaling, with a final increased level of *Caudovirales*, which is observed in IBD patients.^67,77^ Viral dysbiosis in the intestine is consistent with our reports that VDR deletion leads to a higher risk of infection and chronic inflammation.^38,71,78^ Vitamin D metabolites have long been known to support innate antiviral effector mechanisms, including induction of antimicrobial peptides and autophagy.

The diversity and abundance of bacteriophages have been proposed to affect bacterial communities in the gut.^79^ We found a significant correlation between the virome and bacteria altered by VDR status. The enrichment of bacteriophages and related bacteria were consistent, such as *Vibrio* phages and their host *Vibrio cholerae. Bifidobacterium animalis*, one of the bacteria widely used for probiotics in clinical trials,^80,81^ was negatively correlated with BVDV1 and *Vibrio* phage JSF6. The impaired protection of *B. animalis* in the intestinal barrier may further enhance host infection with pathogenic viruses like BVDV1, and intestinal bacteria with bacteriophages like *Vibrio* phage JSF6. Similarly, *Bacteroides acidifaciens*, which was found to have strong protective effects against colitis,^82^ was found to be less abundant and thus negatively correlated with BVDV1. Meanwhile, *Bordetella pseudohinzii* showed a positive correlation with *Vibrio* phage JSF5. As a new member of the genus *Bordetella, B. pseudohinzii* was first identified and isolated from laboratory-raised mice and has now been detected in mouse facilities worldwide.^83^ The infected mice presented elevated numbers of neutrophils in bronchoalveolar lavage fluid and inflammatory signs in histopathology, although no obvious clinical symptoms were shown.^84^ These causative agents may induce more severe inflammation through cooperation with intestinal microbes. Similarly, the abundances of *Vibrio* phage JSF5 and *Bordetella pseudohinzii*, were changed in VDR^ΔPC^ and VDR^ΔLyz^ mice compared to control mice.

The article "Imbalance of the intestinal virome and altered viral-bacterial interactions caused by a conditional deletion of the vitamin D receptor" was published in 2021. Journal: Gut Microbes.

Microbial metabolites are important players in diverse cellular processes and functions. We found marked changes in virus-related metabolites and pathways, such as fatty acid metabolism. It has been suggested that most eukaryotic viruses require lipids or intermediates of lipid synthesis to replicate, and many of them actively induce lipid metabolic pathways to sustention a favorable replication environment.^85^ Pathogenic eukaryotic viruses use lipid droplets as a platform for viral replication, and many non-oncogenic eukaryotic viruses are related to various metabolic alterations during infection, such as glycolysis, nucleotide synthesis, fatty acid biosynthesis and glutaminolysis.^73,86^ This finding may explain our results that many long-chain fatty acid and fatty acid metabolites were increased in VDR^ΔIEC^ and VDR^ΔLyz^ mice.

Although among the most abundant microbes in the gut, phages are also among the least understood.^87^ Using gnotobiotic mice, Hsu et al. found that phage predation not only directly impacts susceptible bacteria but also leads to cascading effects on other bacterial species via interbacterial interactions. Moreover, the shifts in the microbiome caused by phage predation have a direct consequence on the intestinal metabolome as revealed by metabolomic profiling.^36^ We also found that the levels of some phage infection-related metabolites were altered in the conditional VDR knockout mice compared to the control. For example, VDR deletion decreased fecal serine amino acids, which is consistent with a previous study.^36^ Even though various aspects of host central carbon metabolism have been shown to be related to eukaryotic virus infection, several eukaryotic viruses were also found to increase the consumption of key nutrients such as glucose and glutamine and converge on similar metabolic pathways for anabolism,^73^ which was different from our results. It should be mentioned that all these reports are based on host cell metabolic data, while our analysis is based on intestinal microbial metabolites. Furthermore, it is noteworthy that the precise metabolic changes induced by specific viruses are often context-dependent and can vary even within the same viral family or largely depend on the individual host.^73^ However, the regulatory complexity of viral metabolism in chronic diseases is an area of investigation for the future.

The article "Imbalance of the intestinal virome and altered viral-bacterial interactions caused by a conditional deletion of the vitamin D receptor" was published in 2021. Journal: Gut Microbes.

The main limitation of our current study is its descriptive nature. However, it is stage appropriate given the virome/phage field at its early stage. Currently, shotgun metagenomics study of phage and virome as well as their interactions with bacteria is in its infancy stage, an association study is still necessary to explore novel animal models. One goal of this study was to build an appropriate statistical method to analyze the interactions among host, phages, virome and bacteria. The current study did not collect the same fecal samples from the same mice for microbiome and metabolite analysis. It missed an opportunity to identify the metabolic variations in response to the virome and bacteria change from the same host.

In summary, our data have demonstrated that conditional VDR knockout causes changes in the abundance and diversity of the virome and functional changes in viral intestinal receptors, which may further induce intestinal dysbiosis and the risk of infection (Figure 8). We also found that the related fecal metabolites were altered in the mice with tissue-specific deletion, which further confirmed the consequences of dysbiosis. The marked alteration of gut viruses (especially bacteriophages) by VDR status may aid the development of intestinal phage-bacteria or intestinal virus-bacteria therapy against pathobionts.^62,88^ Our study fills the knowledge gaps of how the virome is affected by VDR in a tissue-specific manner. The physiological relevance of these changes will be assessed in the future in digestive disease and infectious models. Notably, there is a growing body of evidence suggesting that VDR activation has a regulatory role in mutualistic intestinal virome-host interactions, and more information on the interactions between the sensing of vitamin D and VDR is needed.^89^

The article "Imbalance of the intestinal virome and altered viral-bacterial interactions caused by a conditional deletion of the vitamin D receptor" was published in 2021. Journal: Gut Microbes.

**Figure 8.** The interrelations of the host, bacteria, and virus. In the host, microbiota, including both bacteria and viruses, could be affected by immune activities, diet, health status and genetic background (e.g., *vdr* gene). In turn, the homeostasis of bacteria and viruses is essential to keep the host healthy. Moreover, bacterial metabolites and viral particles play an important role in host health and the progression of diseases. As one of the viruses, bacteriophages can infect host bacteria and impact bacterial homeostasis. Bacterial products, such as LPS, could be used by the virus for replication. However, the interactions between eukaryotic viruses and bacteria need more study

## Materials and Methods

### Experimental animals

We conditionally deleted vitamin D receptor from intestinal epithelial cells, Paneth cells, and myeloid cells of the mice by crossbreeding VDR^LoxP^ mouse and cre mouse (indicated in Figure 7).

*The genetic background of the mice strains.* The VDR^LoxP^ mice were originally developed by Dr. Geert Carmeliet.^90^ Briefly, the VDR targeting vector was established and electroporated to the R1 embryonic stem cells which was established from a 3.5-day blastocyst produced by crossing two 129 substrains. Then these cells were selected and assessed to get the targeted ES cell clones. Chimeric mice were generated by morula aggregation and bred for germline transmission with Swiss mice. We further backcrossed this strain with C57BL/6 mice for more than 10 generations after arriving our animal facility.

The villin-cre (stock No.: 004586) transgenic mice were purchased from The Jackson Laboratory (Bar Harbor, ME, USA), which were generated with C57BL/6 background, based on the information from JAX. Briefly, the designed VilCre transgene was injected into the pronuclei of fertilized C57BL/6 J x SJL/J mouse eggs. Several founder animals were bred to C57BL/6 mice for germline transmission, and founder line 997 was established. The Vil1-Cre 997 mice were subsequently backcrossed to C57BL/6 mice for five generations, and were further crossed to C57BL/6 J at least once to establish the colony after arriving at The Jackson laboratory.

The Lyz-cre mice were purchased from The Jackson Laboratory (stock No.: 004781). Briefly, the targeting vector was designed and electroporated into 129P2/OlaHsd-derived E14.1 embryonic stem (ES) cells. Correctly targeted ES cells were injected into blastocysts. The resulting chimeric animals were crossed to C57BL/6 mice for at least six generations prior to sending to The Jackson Laboratory Repository.

The Defa6-cre mice were provided by Dr. Richard Blumberg.^71,91^ This Paneth cell-specific Defa6-cre mouse strain was generated by injecting the designed plasmid into the pronuclear of C57BL/6 mice.

The article "Imbalance of the intestinal virome and altered viral-bacterial interactions caused by a conditional deletion of the vitamin D receptor" was published in 2021. Journal: Gut Microbes.

VDR^ΔIEC^, VDR^ΔPC^ and VDR^ΔLyz^ mice were obtained by crossing the VDR^LoxP^ mice with villin-cre, Defa6-cre and Lyz-cre mice, respectively. All the mice used in this study were with C57BL/6 genetic background by generating or crossing with C57BL/6 mice.

*Breeding method.* Conditional knockout (KO) mice were derived from heterozygous mating pairs such that conditional KO mice came from the same litter. The same breeding method was used for the VDR^LoxP^ mice. All the animals are asymptomatic when the samples were collected.^37,71,92^ The breeders were setup at the similar time to get enough knockout and control mice with the similar age for sample collection.

*Biosecurity and routine pathogen screening.* All the animals were housed in the Biologic Resources Laboratory (BRL) at the University of Illinois at Chicago (UIC) and utilized in accordance with the UIC Animal Care Committee (ACC) and Office of Animal Care and Institutional Biosafety (OACIB) guidelines. The animal work was approved by the UIC Office of Animal Care (ACC15-231, ACC17-218, and ACC18-216).

Mice from the approved sources, such as JAX, are commercial vendors who conduct regular and comprehensive colony health monitoring, exclude specific murine pathogens as identified by the veterinary staff, practice high management standards, and ship animals directly via a dedicated ground transportation network. Sources that do not meet these criteria are considered non-approved vendors. The UIC BRL veterinary staff did quarantine or rederivation after the indicated mice were shipped to UIC.

Many methods are used to maintain biosecurity within the UIC animal facilities. Firstly, the health monitoring program for mice utilizes sentinel animals to assess the pathogen status of UIC colonies. Sentinel mice are tested quarterly by serology, PCR, and parasitology. Comprehensive serologic testing of sentinel mice is performed annually. Secondly, animal housing is used to control the spread of infectious agents. The mice are housed in sterilized static microisolator cages, which provide an effective barrier to the entry and spread of microbial agents. Another means to decrease pathogen exposure and spread is through disinfection of all shared-use equipment and space prior to use. In doing so, it helps ensure animal health which in turn minimizes confounding variables to research models and maintain the specific pathogen status of animal colonies.

The BRL veterinary staff monitors the health status of the institution’s rodent colonies through a dirty bedding sentinel program. Sentinel animals within a room are exposed weekly to dirty bedding from a designated section of research animal cages. Dirty bedding sentinels are most effective at detecting pathogens transmitted primarily by fecal-oral contamination. This method of health surveillance detects agents without the need to directly test research animals. Sentinel animals are tested quarterly for murine pathogens including endo and ectoparasites. The information obtained from sentinel animal health assessments is used for the early detection of a disease outbreak, to generate health reports for animals being exported, and to maintain a high level of quality control within animal rooms and facilities. The personal protective equipment for operators and strategies for the animals to maintain biosecurity within the UIC animal facilities were followed according to the animal facility guidelines.^93^

The article "Imbalance of the intestinal virome and altered viral-bacterial interactions caused by a conditional deletion of the vitamin D receptor" was published in 2021. Journal: Gut Microbes.

*Study design and power analysis.*The animals (male and female; aged 6 to 8 weeks) studied in this research include three conditional VDR-knockout (VDR^ΔIEC^, VDR^ΔPC^ and VDR^ΔLyz^) and control VDR^LoxP^ mice. Power analysis suggested that the number of 10 animals used in each group can provide sufficient power to detect the differences among groups for metagenomic analysis. All the animals were randomly assigned to each group. All the animals used in our study were apparently healthy when the fecal sample collection was performed.

## Real-time quantitative PCR

Total RNAs were extracted from colon epithelial cells of four genotype mice of VDR^LoxP^, VDR^ΔIEC^, VDR^ΔPC^ and VDR^ΔLyz^, using TRIzol reagent (15,596–018, Life technologies, Carlsbad, CA, USA). RNAs were first reverse-transcribed into cDNA with the iScript cDNA synthesis kit (1,708,890, Bio-Rad, Hercules, CA, USA) according to the manufacturer’s manual. The CTFX 96 Real-time system (Bio-Rad, Hercules, CA, USA) and SYBR Green Supermix (172–5120, Bio-Rad, Hercules, CA, USA) were used for the quantitative real-time PCR with the RT-cDNA reaction products according to the manufacturer’s directions. All expression levels were normalized to β-actin levels of the same sample. Percent expression was calculated as the ratio of the normalized value of each sample to that of the corresponding untreated ones. All real-time PCR reactions were performed in triplicate. Optimal primer sequences target for PRRs were obtained from Primer Bank^94^ (http://pga.mgh.harvard.edu/primerbank/) as listed in Table 1.

## Fecal sample collection and shotgun metagenomic sequencing

We used whole-genome shotgun sequencing to sequence fecal samples. Fresh fecal samples from each group (VDR^LoxP^: male n = 3 and female n = 7; VDR^ΔIEC^: male n = 5 and female n = 5; VDR^ΔPC^: male n = 5 and female n = 5; VDR^ΔLyz^: male n = 5 and female n = 5) were collected from the colon and placed into the sterile tubes. The samples were kept at low temperature with dry ice and were sent to the University of Illinois at Chicago Research Resources Center for genomic sequencing. The DNAs of samples were extracted using DNeasy Power Fecal Kit (12,830, Qiagen, Hilden, Germany) based on manufacturer’s instructions with a slight modification. The samples were heated at 65°C for 10 min before homogenizing with FastPre-24 5 G bead-beating device (MP Biomedicals, Solon, OH, USA) at 6 m/s for 40 s. These genomic DNAs were fragmented into relatively small pieces (generally 250–600 bp fragments) before sequencing. Sequencing was performed using a Illumina HiSeq system, as in our previous publications.^69,71^ Following quality checking, filtering the reads, removing noisy sequences, and metagenomic assembly,^95^ the resulting assemblies were filtered to exclude contigs shorter than 1,000 nucleotides and all remaining set of DNA reads (or contigs) were classified with Centrifuge,^96^ an efficient metagenomic classifier capable of indexing the entirety of nucleotide (nt). Next, the taxonomic annotation of each contig (genes) was obtained by searching for the comprehensive NCBI GenBank non-redundant nucleotide database (as described in https://merenlab.org/2016/06/18/importing-taxonomy^97^). After removing the identical sequences with ≥99% identity of each other to make it nonredundant, 289,629,756 readable sequences were yielded in 40 studied samples with an average of 7,240,744 reads per sample. Of these sequences, a total of 100,013,480 reads were taxonomic alignments with an average of 2,500,337 reads per sample.

The article "Imbalance of the intestinal virome and altered viral-bacterial interactions caused by a conditional deletion of the vitamin D receptor" was published in 2021. Journal: Gut Microbes.

## Metabolite sample preparation and metabolomic data analysis

*Sample preparation and process.* As in our pervious report,^69^ metabolite profiling was performed on Metabolon platform (Metabolon, Inc., Durham, NC, USA). Briefly, fecal samples from a different set of animals from each group (VDR^LoxP^: male n = 6 and female n = 10; VDR^ΔIEC^: male n = 8 and female n = 9; VDR^ΔLyz^: male n = 5 and female n = 5)^69^ were maintained at −80°C and were prepared using the automated MicroLab STAR® system from Hamilton Company. Several recovery standards were added prior to the first step in the extraction process for QC purposes. The proteins were precipitated with methanol under vigorous shaking for 2 min (Glen Mills GenoGrinder 2000) followed by centrifugation to remove protein, dissociate small molecules bound to protein or trapped in the precipitated protein matrix, and to recover chemically diverse metabolites. Next, samples were placed on a TurboVap® (Zymark) briefly to remove the organic solvent. The sample extracts were stored overnight under nitrogen before preparation for analysis. The resulting extract was divided into five fractions for analysis by four methods using Ultrahigh Performance Liquid Chromatography-Tandem Mass Spectroscopy (UPLC-MS/MS) (see details in the bioinformatic analysis below) and one for backup.

The article "Imbalance of the intestinal virome and altered viral-bacterial interactions caused by a conditional deletion of the vitamin D receptor" was published in 2021. Journal: Gut Microbes.

*Bioinformatic analysis of metabolomic data.* Bioinformatic analysis was performed using the Metabolon informatic system (the LAN backbone, and a database server running Oracle 10.2.0.1 Enterprise Edition), which consists of four major components, including the Laboratory Information Management System (LIMS), the data extraction and peak-identification software, data processing tools for QC and compound identification, and a collection of information interpretation and visualization tools for use by data analysis. The hardware and software foundations for these informatic components were the LAN backbone and a database server running Oracle 10.2.0.1 Enterprise Edition.

*Data extraction and compound identification*. After raw data extraction, peak-identification and QC process using Metabolon’s hardware and software in its platform (https://www.metabolon.com), compounds were identified by comparison to library entries of more than 3300 currently commercially available purified standard compounds or recurrent unknown entities. Metabolon maintains a library based on authenticated standards that contains the retention time/index (RI), mass to charge ratio (*m/z)*, and chromatographic data (including MS/MS spectral data) on all molecules present in the library. Furthermore, biochemical identifications are based on three criteria: retention index within a narrow RI window of the proposed identification, accurate mass match to the library ± 10 ppm, and the MS/MS forward and reverse scores between the experimental data and authentic standards.

*Metabolite quantification and data normalization*. Peaks were quantified using area-under-the-curve. A data normalization step was performed to correct variation resulting from instrument inter-day tuning differences as necessary or for purposes of data visualization. Additionally, biochemical data were normalized to other factors (e.g., cell counts, total protein as determined by Bradford assay, and osmolality) to account for differences in metabolite levels due to differences in the amount of material present in each sample.

## Statistical analysis

All the tests as specified in related analysis performed in study were two-sided. A *P*-value ≤0.05 was considered statistically significant. For a large number of tests, the *P*-values were adjusted to account for false positives using the False Discovery Rate (FDR)^98^ and the q-value (FDR-corrected *p*-value) ≤0.05 was reported to be significant. For all the data, we ran Shapiro-Wilk test to determine whether parametric ANOVA or non-parametric Kruskal-Wallis test is used to group comparisons.

The article "Imbalance of the intestinal virome and altered viral-bacterial interactions caused by a conditional deletion of the vitamin D receptor" was published in 2021. Journal: Gut Microbes.

Alpha (within-sample) diversity (e.g., Shannon diversity) measures the number (richness) and/or distribution (evenness) of species within a single sample, while beta (between-sample) diversity (e.g., Bray-Curtis dissimilarity) measures the differences of microbial composition in one sample compared to another^41^ For the metagenomic sequencing data, the raw read counts were normalized to Counts Per Million (CPM). Shannon diversity was used to examine the diversity of the gut microbiome in conditional VDR KO and control mice and the differences between groups were tested with Kruskal-Wallis test.

Bray-Curtis dissimilarity index was used to detect the differences or dissimilarities among studied groups. We first performed principal coordinate analysis (PCoA) to visualize the Bray-Curtis dissimilarities among groups. Next, we performed the nonparametric PERMANOVA to evaluate whether the group (VDR^ΔIEC^, VDR^ΔPC^, and VDR^ΔLyz^ mice vs. VDR^LoxP^ mice) has a significant effect on overall gut microbiota composition. Next, we performed pairwise PERMANOVA using RVAideMemoire package. Finally, we conducted analysis of similarity (ANOSIM), another nonparametric procedure, based on a permutation test for rank dissimilarities among between- and within-groups to confirm the hypothesis testing results from those of PERMANOVA and obtained the pairwise-comparison results. The Spearman correlation analysis of viruses and bacteria was performed via the Hmisc package.^99^

The statistical analysis of metabolites was performed using Welch’s two-sample *t*-test on log transformed data. Welch’s two-sample *t*-test is used to test whether two unknown means are different from two independent populations, which enables unequal variances and has an approximate*t*-distribution with degrees of freedom estimated using Satterthwaite’s approximation. The log_2_ fold-changes were reported as the effect sizes in comparisons between groups.^100^ The statistical analyses for microbiome and metabolomic data were performed using R,^101^ R packages of ampvis2, microbiome, phyloseq and vegan,^41^ as well as ggplot2^102^ and ggpubr packages.^103^

## Supplementary Material

Supplemental Material

## List of abbreviations

*ATG16L1*: Autophagy Related 16 Like 1

BVDV 1: Bovine viral diarrhea virus 1

CD: Crohn’s disease

CLEC4L: C-type lectin domain family 4

CLRs: C-type lectin receptors

COVID19: coronavirus disease 2019

CRC: Colorectal cancer

HBGA: human blood group antigen

IBD: Inflammatory bowel disease

LPS: Lipopolysaccharide

TLR: Toll-like receptor

NOD: nucleotide-binding oligomerization domain

NLRs: nucleotide-binding oligomerization domain-like receptor

PCoA: performed principal coordinate analysis

PERMANOVA: nonparametric permutational multivariate analysis of variance

PRR: Pattern recognition receptors

UC: Ulcerative colitis

The article "Imbalance of the intestinal virome and altered viral-bacterial interactions caused by a conditional deletion of the vitamin D receptor" was published in 2021. Journal: Gut Microbes.

## Declarations

- Ethics approval and consent to participate: The animal work was approved by the Office of Animal Care and Institutional Biosafety (OACIB) and UIC Animal Care Committee (ACC) with accession number of ACC15-231, ACC17-218, and ACC18-216.·  The contents do not represent the views of the United States Department of Veterans Affairs or the United States Government.

No human study. All animal studies were performed following ACC guidelines at the University of Illinois at Chicago (UIC), IL, U.S.A.

Consent for publication: Not applicable.

Availability of data and material: the metagenomic data was submitted to Github:

https://github.com/jileiz/Shotgun-Virome
